# Prognostic Analysis of LncRNA MCM3AP-AS1 in Colorectal Cancer and the Mechanism of Its Effect on Tumor Cell Activity

**DOI:** 10.1155/2022/1616370

**Published:** 2022-09-19

**Authors:** Qi Song, Jinsuo Gao, Jinzhu Yang, Subash C. B. Gopinath, Lei Shen

**Affiliations:** ^1^Department of Oncology, Anhui Medical University, Hefei Third Clinical College, The Third People's Hospital of Hefei, Hefei, Anhui 230022, China; ^2^Faculty of Chemical Engineering Technology, Universiti Malaysia Perlis (UniMAP), 02600 Arau, Perlis, Malaysia; ^3^Institute of Nano Electronic Engineering, Universiti Malaysia Perlis (UniMAP), Kangar 01000, Perlis, Malaysia; ^4^Micro System Technology, Centre of Excellence (CoE), Universiti Malaysia Perlis (UniMAP), Arau 02600, Pauh Campus, Perlis, Malaysia

## Abstract

To determine the clinical prognostic significance of lncRNA MCM3AP-AS1 in colorectal cancer (CRC) and its preliminary mechanism, 43 CRC patients and 48 healthy individuals were analyzed. Peripheral blood MCM3AP-AS1 was quantified via qRT–PCR in CRC patients at admission and 2 h after surgery and in healthy individuals. Human colon cancer cells (HCT116 and SW480) were transfected with shRNAs targeting upregulation of MCM3AP-AS1 expression (named as sh-MCM3AP-AS1 group) and corresponding negative RNAs (named as sh-MCM3AP-AS1 group). Additionally, the cells were then treated either with 50 mM of the VEGF-specific inhibitor PTK787 (Selleck, USA) (named as inhibition group) or normal saline as a control (named as control group). Before therapy, CRC patients presented a higher MCM3AP-AS1 level than healthy individuals (*P* < 0.05), and the sensitivity and specificity of MCM3AP-AS1 in predicting the occurrence of CRC were 65.12% and 83.33%, respectively (*P* < 0.001). After therapy, CRC patients presented a decrease in MCM3AP-AS1 levels, and recurrence was higher in patients who died (*P* < 0.05). Additionally, the high MCM3AP-AS1 expression group presented a higher mortality than the low MCM3AP-AS1 expression group (*P* < 0.05). In an *in vitro* assay, CRC cells showed a higher MCM3AP-AS1 level than CCD-18Co cells, and the sh-MCM3AP-AS1 group presented decreased cell proliferation and invasiveness, whereas the levels apoptosis-associated proteins were increased (*P* < 0.05). Moreover, the VEGF and VEGFR2 mRNA levels were increased in CRC cells, and VEGF/VEGFR2 pathway-associated proteins were inhibited in the sh-MCM3AP-AS1 group (*P* < 0.05). Moreover, treatment with PTK787 decreased cell proliferation and invasivness but increased the levels of apoptosis-associated proteins (*P* < 0.05).

## 1. Introduction

Colorectal cancer (CRC) is a common malignant tumor that originates from intestinal sites, including the rectum, sigmoid colon, and ascending colon [1]. Over 1.8 million new patients were diagnosed with CRC in 2018 worldwide [2]. In recent years, the incidence of CRC has increased, and young people are increasingly afflicted [2, 3]. In the early phase, CRC lacks characteristic clinical symptoms. Consequently, it usually is diagnosed at the middle or late stage once clear hematochezia and intestinal obstruction occur, and the risks of infiltration and metastasis at this stage are high [4]. One survey indicated that advanced CRC has a 5-year mortality rate of over 40%, second only to that of lung cancer (LC) [5, 6]. Therefore, CRC has long been the focus of clinical research to identify novel and effective and timely diagnosis and treatment methods and improve prognosis.

In recent, lncRNAs have been confirmed to strongly regulate the activities of various cells. Moreover, the development of tumors is related to the invasiveness and proliferation of tumor cells [7–9]. A growing number of studies have noted that fully understanding the impacts of lncRNAs on tumor cells may lead to breakthroughs in the future diagnosis and treatment of tumors. lncRNA MCM3AP-AS1 (MCM3AP-AS1) is an lncRNA discovered in recent years that was first confirmed to have abnormal expression in spongioblastoma [10]. Its regulation of pancreatic cancer and LC cells has gradually captured clinical attention [11, 12]. Recently, Lu et al. found abnormal MCM3AP-AS1 lncRNA expression in CRC during screening [13]. A follow-up study preliminarily confirmed that MCM3AP-AS1 was associated with CRC [14] Thus, MCM3AP-AS1 may be of great significance for the future diagnosis and treatment of CRC. However, as associated research is relatively rare at the current stage, the clinical mechanism underlying the role of MCM3AP-AS1 in CRC requires further exploration.

Accordingly, this study analyzed the effect of MCM3AP-AS1 on the prognosis of CRC patients by detecting the expression of MCM3AP-AS1 in CRC and explored the preliminary mechanism of CRC through *in vitro* experiments. This study was designed to confirm the clinical role and significance of MCM3AP-AS1 in CRC, lay the foundation for subsequent related research, and provide novel ideas and directions for the future clinical diagnosis and treatment of CRC.

## 2. Materials and Methods

### 2.1. Data about Patients

In total, 43 CRC patients admitted to the Third People's Hospital of Hefei between July 2020 and October 2020, and 48 healthy individuals identified during the same time period were enrolled and prospectively analyzed. This experiment was approved by the Ethics Committee of our hospital. All participants signed informed consent forms.

### 2.2. Inclusion and Exclusion Criteria

The inclusion criteria for patients were as follows: patients confirmed to have CRC by biopsy in the pathology department, patients whose pathogenic site was in the right or left colon, patients whose histologic type was adenocarcinoma, patients in the early phase in terms of pathological stage, and patients >18 years old. The exclusion criteria for patients were as follows: cases complicated by multiple tumors, cardiovascular or cerebrovascular diseases, infectious diseases, autoimmune diseases, or organ dysfunction; pregnant or lactating patients; referred patients; and patients who received cancer therapy within the half year before admission. The inclusion criteria for healthy individuals were as follows: individuals whose physical examination results were all normal, individuals without a history of major diseases, and individuals >18 years old.

### 2.3. Data about Cells

Human colon cancer cells (HCT116 and SW480) and human normal colon cells (CCD-18Co) were provided by ATCC. HCT116 and CCD-18Co cells were incubated with medium (90% glutamine and 10% FPS), and SW480 cells were subjected to incubation (37°C) in high-sugar medium (90% glutamine and sodium pyruvate and 10% FPS, matching cell medium, ATCC) under 5% CO_2_.

### 2.4. Blood Sample Collection

After admission, CRC patients were all treated with radical tumor resection by the same senior surgical team at our hospital. Fasting venous peripheral blood (4 mL) was sampled from each CRC patient at admission (before therapy) and 2 h after surgery (after therapy) and from each healthy individual at admission. The blood samples were collected in coagulation-promoting tubes, followed by 20 min of centrifugation (1505 × *g*) after coagulation to obtain serum. The serum was stored in an -80°C freezer for later assays.

### 2.5. Cell Transfection

The original culture medium of HCT116 and SW480 cells was removed, and the cells were washed with PBS, followed by the addition of trypsin (ThermoFisher, USA) for cell digestion. Under a microscope (Phoenix XSP-06-1600X), most of the trypsin was removed once the cells had detached, leaving approximately 0.5 mL of supernatant. The cells were then placed in an incubator for digestion and removed after approximately 3 minutes. HCT116 and SW480 cells in the log phase were collected, followed by trypsinization to prepare a cell suspension, and the suspension was then transferred to a 12-well plate. Cells at a cell confluency of 70-80% were transfected with shRNAs targeting upregulation of MCM3AP-AS1 expression (named as sh-MCM3AP-AS1 group) and corresponding negative RNAs (named as sh-MCM3AP-AS1 group). The cells were transfected with Lipofectamine 2000 (Thermo Fisher, USA) according to the manufacturer's protocol and subsequently incubated for 48 h (37°C). Additionally, the cells were then treated either with 50 mM of the VEGF-specific inhibitor PTK787 (Selleck, USA) (named as inhibition group) or normal saline as a control (named as control group).

### 2.6. qRT–PCR

Total RNA from blood or cells obtained by TRIzol kit (Thermo Fisher, USA), followed by purity verification with a UV spectrophotometer (Multiskan SkyHigh, Thermo Fisher, USA). The RNA was then reverse transcribed to obtain cDNA according to the guidelines of the reverse transcription kit (Thermo Fisher, USA) under the following reaction conditions: 95°C/60 s, followed by 40 cycles of 95°C/15 s, 60°C/34 s, and 72°C/45 s. The primer sequences are summarized in Table 1 (the primer sequences were designed and constructed by Beijing Tsingke Biotechnology Co., Ltd.). MCM3AP-AS1 uses GAPDH as internal control; VEGF and VEGFR2 use *β*-actin as internal control; the relative expression was calculated with the 2^−△△ct^ method.

### 2.7. MTT Assay

Trypsinized (Thermo Fisher, USA) cells whose concentration was adjusted to 3 × 10^4^ cells/mL were transferred to a 96-well plate (200 *μ*L/well, Abcam, USA). After 0, 24, 48, and 72 h, MTT reagent (20 *μ*L/well) was added to each well, followed by 2 h of continuous incubation, and the optical density (490 nm) was then determined with an enzyme reader.

### 2.8. Transwell Assay

Diluent (40 *μ*L/well) and 0.25% trypsin were added to the upper and lower compartments of the Transwell insert (Sigma–Aldrich, USA), respectively. After digestion, FBS-free cells at the log phase (5 × 10^4^ cells/mL) in the lower compartment were mixed. After 24 h of incubation, the cells were washed three times with PBS, and paraformaldehyde (Sigma–Aldrich, USA) treatment for 10 min was used to fuse and immobilize membrane-penetrating cells. The cells were stained with 0.1% crystal violet. Cells in 5 randomly selected visual fields were evaluated under a microscope.

### 2.9. Western Blot Assay

The cells were digested with trypsin, washed three times with PBS solution, added with an appropriate amount of protein extract (Beijing Soleibo Technology Co., Ltd., China), and shaken in an ice bath for 15 min. After centrifugation (10,000 × g, 4°C) for 20 min, the supernatant was collected and aliquoted into EP tubes, followed by protein purity determination via the BCA kit (Abcam, USA) method. Afterward, 30 *μ*g of protein was subjected to SDS–PAGE (Thermo Fisher, USA) and transferred onto a PVDF membrane (Sigma–Aldrich, USA), followed by 2 h of immersion in 5% skim milk and subsequent overnight incubation with antibodies against Bax (1 : 1000), Caspase-3 (1 : 1000), and *β*-actin (1 : 1000) (TaKaRa, Japan) at room temperature. The next day, the membranes were washed three times with TBST, followed by a 1 h incubation with the secondary antibody (1 : 2000). Subsequently, the membranes were also washed three times with TBST, followed by exposure and development. A gel imaging system (iBright, Thermo Fisher, USA) and the ImageJ software (National Institutes of Health) were used to analyze the gray value and calculate the relative protein expression.

### 2.10. Follow-Up

CRC patients were followed up for 1 year via hospital reexamination, and their survival and recurrence within 1 year were both recorded.

### 2.11. Statistical Analyses

The SPSS 22.0 software (IBM, USA) was used to analyze the obtained results. Measurement data (^−^*χ* ± *s*) were analyzed using the independent-samples T test, one-way ANOVA, and LSD post hoc test. Count data [*n* (%)] were analyzed using the chi-squared test. The Kaplan–Meier method was used to analyze the survival rate, and the log-rank test was to compare survival rates. *P* < 0.05 implies a notable difference.

## 3. Results

### 3.1. Clinical Value of MCM3AP-AS1

CRC patients before therapy presented a higher MCM3AP-AS1 level than healthy individuals at admission (*P* < 0.05, Figure 1(a)), indicating that MCM3AP-AS1 is highly expressed in CRC. According to the ROC curve-based analysis, MCM3AP-AS1>6.175 had a sensitivity of 65.12% and specificity of 83.33% in predicting the occurrence of CRC (*P* < 0.001, Figure 1(b)).

### 3.2. Prognostic Value of MCM3AP-AS1

The expression level of MCM3AP-AS1 in CRC patients after treatment was significantly lower than before treatment (*P* < 0.05, Figure 2(a)). At the 1-year follow-up, 6 patients had died and 8 patients had experienced recurrence. The expression level of MCM3AP-AS1 in patients who died after treatment was higher than that in patients who survived (*P* < 0.05, Figure 2(b)), and the expression level of MCM3AP-AS1 was also higher in patients with disease recurrence after treatment than in patients without disease recurrence (*P* < 0.05, Figure 2(c)). According to the ROC curve-based analysis, an MCM3AP-AS1 level>6.535 after therapy had a sensitivity of 83.33% and a specificity of 83.78% in predicting the death of patients (*P* < 0.05, Figure 2(d)), and an MCM3AP-AS1 level>5.890 after therapy had a sensitivity of 100.0% and a specificity of 54.29% in predicting the recurrence of patients (*P* < 0.05, Figure 2(e)). Based on this cutoff value, the patients were assigned to two groups: the high MCM3AP-AS1 expression group (MCM3AP-AS1>6.105 after therapy) or the low MCM3AP-AS1 expression group. The results showed that the former group had a notably higher mortality than the latter group (36.36% *vs.* 6.25%, *P* < 0.05, Figure 2(f)).

### 3.3. Analysis of MCM3AP-AS1 Based on Database

In the ENCORI database (https://starbase.sysu.edu.cn/index.php), a high MCM3AP-AS1 level was found in tumors, including cholangiocarcinoma, liver cancer, and gastric cancer, and the increase in MCM3AP-AS1 also indicated an elevation in the mortality of tumors, including kidney cancer, liver cancer, and colon adenocarcinoma (Figure 3).

### 3.4. Effect of MCM3AP-AS1 Silencing on the Proliferation and Invasion of CRC Cells

The MCM3AP-AS1 expression levels in HCT116 and SW480 cells, which were notably higher than that in CCD-18Co cells (*P* < 0.05, Figure 4(a)). Additionally, the abilities of HCT116 and SW480 cells to proliferate 72 h after sh-MCM3AP-AS1 OD values were (0.43 ± 0.04) and (0.44 ± 0.05), respectively. The OD values of the NC-MCM3AP-AS1 group were (0.57 ± 0.05) and (0.62 ± 0.05), respectively. It can be seen that the cell proliferation ability of the sh-MCM3AP-AS1 group was lower than that of the NC-MCM3AP-AS1 group (*P* < 0.05, Figures 4(b) and 4(c)). Transwell experiments were adopted to detect the influence of MCM3AP-AS1 on the invasiveness of CRC cells, and the staining results are shown in Figure 4(d). In HCT116 and SW480 cells, the numbers of invading cells in sh-MCM3AP-AS1 group, which were also lower than the number of invading cells in the NC-MCM3AP-AS1 group (*P* < 0.05, Figure 4(e)).

### 3.5. Effect of Interference with MCM3AP-AS1 on CRC Cell Apoptotic Protein

Western blotting was used to detect Bax and Caspase-3 protein expression in CRC and analyze the effect of MCM3AP-AS1 on CRC cell apoptosis. The protein imprinting map of HCT116 cells is shown in Figure 5(a); the Bax and Caspase-3 protein expression levels in the sh-MCM3AP-AS1 group, which were higher than those in the NC-MCM3AP-AS1 group (*P* < 0.05, Figure 5(b)). The Western blot of SW480 cells is shown in Figure 5(c); the expression levels of Bax and Caspase-3 proteins in the sh-MCM3AP-AS1 group in SW480 cells, which were higher than those in the NC-MCM3AP-AS1 group (*P* < 0.05, Figure 5(d)). According to these results, we can know that Bax and Caspase-3 proteins are highly expressed in the sh-MCM3AP-AS1 group, indicating that the apoptotic ability of cells is enhanced.

### 3.6. Impacts of MCM3AP-AS1 on the VEGF/VEGFR2 Pathway

The expression levels of VEGF and VEGFR2 mRNA in HCT116 cells were 2.07 ± 0.30 and 2.14 ± 0.12, respectively, and the expression levels of VEGF and VEGFR2 mRNA in SW480 cells were 1.82 ± 0.29 and 1.82 ± 0.13, respectively. The expression levels of VEGF and VEGFR2 in HCT116 and SW480 cells were higher than those in CCD-18Co cells (*P* < 0.05, Figure 6(a)). The levels of VEGF and VEGFR2 mRNA in the sh-MCM3AP-AS1 group in HCT116 cells, which were lower than those in the NC-MCM3AP-AS1 group (*P* < 0.05, Figure 6(b)). The levels of VEGF and VEGFR2 mRNA in the sh-MCM3AP-AS1 group in SW480 cells, which were lower than those in the NC-MCM3AP-AS1 group (*P* < 0.05, Figure 6(c)). Western blotting was used again to detect the expression of the VEGF/VEGFR2 pathway-related proteins VEGF, t-VEGFR2, and p-VEGFR2 for verification. The results of protein detection in HCT116 cells are shown in Figure 6(d). The expression levels of VEGF, t-VEGFR2, and p-VEGFR2 in the sh-MCM3AP-AS1 group, which were lower than those in the NC-MCM3AP-AS1 group (*P* < 0.05, Figure 6(e)). The results of protein detection in SW480 cells are shown in Figure 6(f). The expression levels of VEGF, t-VEGFR2, and p-VEGFR2 in the sh-MCM3AP-AS1 group, which were lower than those in the NC-MCM3AP-AS1 group (*P* < 0.05, Figure 6(g)). It can be observed that the Western blot results are also consistent with the PCR results, indicating that downregulating the expression of MCM3AP-AS1 will inhibit the VEGF/VEGFR2 signaling pathway.

### 3.7. Effect of Inhibiting the VEGF/VEGFR2 Pathway on the Proliferation and Invasiveness of CRC Cells

In HCT116 cells, OD value at 72 h was 0.42 ± 0.06 in the inhibition group; the OD value of the control group at 72 h was (0.57 ± 0.05). After the comparison, it was found that the cell proliferation ability of the inhibition group was lower than that of the control group (*P* < 0.05, Figure 7(a)). In SW480 cells, OD value at 72 h was 0.42 ± 0.03 in the inhibition group; the OD value of the control group at 72 h was (0.61 ± 0.03); the cell proliferation ability of the inhibition group was also lower than that of the control group (*P* < 0.05, Figure 7(b)). The Transwell experiment was used to detect the effect of the VEGF/VEGFR2 pathway on the invasiveness of CRC cells, and the staining results are shown in Figure 7(c). In HCT116 and SW480 cells, 57.67 ± 6.03 and 62.00 ± 4.36 cells had invaded in the inhibition group, respectively, and these numbers were also lower than the numbers observed in the control group (*P* < 0.05, Figure 7(d)). It indicated that the cell invasion ability of the inhibition group was also lower than that of the control group.

### 3.8. Effect of Inhibiting the VEGF/VEGFR2 Pathway on Apoptotic Proteins in CRC Cells

Western blotting was used to detect Bax and Caspase-3 protein expression in CRC. The Western blot map of HCT116 cells is shown in Figure 8(a); the expression levels of Bax and Caspase-3 proteins in the inhibition group, which were higher than those in the control group (*P* < 0.05, Figure 8(b)). The Western blot map of SW480 cells is shown in Figure 8(c); the protein expression levels of Bax and Caspase-3 in the inhibition group in SW480 cells, which were higher than those in the control group (*P* < 0.05, Figure 8(d)). These data tell us that after inhibition of VEGF/VEGFR2 signaling pathway, the ability of cells to apoptotic rate is enhanced.

## 4. Discussion

Currently, CRC poses a growing threat [15], and fully understanding its pathogenic mechanism may be the key to preventing, diagnosing, and treating it in the future. As a hotspot in clinical research, lncRNAs can strongly regulate cells and are also detectable in tissues, blood, and cells [16, 17]. Confirming the role of MCM3AP-AS1 in CRC allows the adoption of MCM3AP-AS1 as a diagnostic marker of tumors to improve the early detection rate. In addition, disease progression can be judged based on MCM3AP-AS1 to help clinicians take effective intervention measures as soon as possible. Targeted therapy with MCM3AP-AS1 may be more effective and safer than current surgery, radiotherapy, and chemotherapy [18, 19].

In this assay, we first quantified serum MCM3AP-AS1 in CRC patients and healthy individuals and identified high MCM3AP-AS1 expression among CRC patients. Chen et al. [20] reported that MCM3AP-AS1 was also highly expressed in breast cancer, which suggests that the expression of MCM3AP-AS1 is consistent in a variety of tumor diseases and corroborates the results of this experiment. A subsequent ROC curve-based analysis showed that the sensitivity and specificity of MCM3AP-AS1 in predicting CRC occurrence were 69.72% and 76.86%, respectively. Currently, tumor markers that are commonly adopted in clinical scenarios include CEA and CA199, which are sensitive to tumor reactions but have low specificity [21]. The analysis results of MCM3AP-AS1 can compensate for the shortcomings of traditional cancer markers. We inferred that the early detection rate of CRC can be effectively increased by the joint detection of MCM3AP-AS1 and cancer markers in the future. In addition, we found a decrease in MCM3AP-AS1 in CRC patients after therapy and discovered its strong association with the survival and recurrence of CRC patients. Based on the survival curve, high MCM3AP-AS1 expression after therapy denoted an increased risk of death of patients, which once again emphasized the great potential value of MCM3AP-AS1 in CRC. At present, a reliable evaluation index for the prognosis of tumor diseases is lacking, but the application of MCM3AP-AS1 can greatly improve the ability of clinicians to evaluate CRC, intervene in time, and provide a more reliable guarantee for the prognosis of patients. Similarly, Wang et al. [22] showed that MCM3AP-AS1 has the potential to become a prognostic marker of liver cancer, which also suggests that the future application of MCM3AP-AS1 in tumor diseases may not only be limited to CRC but also have potential evaluation significance for other tumors. Moreover, to further verify the expression of MCM3AP-AS1, its expression in tumors, including cholangiocarcinoma, was also explored in an online database and found to be highly expressed [22], which once again verifies the accuracy of the experimental results and confirms the expression of MCM3AP-AS1 in CRC. To verify the mechanism of MCM3AP-AS1 in CRC, we carried out an *in vitro* assay and found that suppressing MCM3AP-AS1 strongly accelerated the apoptosis of CRC cells and improve their growth and invasiveness, which suggested the oncogenic role of high MCM3AP-AS1 expression in CRC. In oral squamous cell carcinoma, high MCM3AP-AS1 expression can also promote the growth of tumor cells, which supports the conclusion of our study [23] and further confirms the effect of MCM3AP-AS1 on tumor diseases. According to related research, Yu et al. identified the function of MCM3AP-AS1 in regulating the activity of endometrial cancer cells via VEGF [24]. VEGF, a crucial link in the development of tumor diseases, has also been verified to promote the angiogenesis of CRC by activating its receptor, VEGFR2 [25]. Accordingly, we preliminarily inferred a possible association between the MCM3AP-AS1 and VEGF/VEGFR2 pathways in CRC. We experimentally identified notable decreases in VEGF and VEGFR2 in CRC cells, which verified their involvement in the development of CRC and was consistent with the results of previous studies [26, 27]. In addition, VEGF and VEGFR2 expression decreased in the sh-MCM3AP-AS1, which indicated that silencing MCM3AP-AS1 could also inhibit the activation of the VEGF/VEGFR2 pathway. Finally, PTK787 treatment inhibited the invasiveness and proliferation of CRC cells and increased the levels of apoptosis-associated proteins, suggesting that suppressing the VEGF/VEGFR2 pathway could also hinder the development of CRC cells. The above experimental results indicate that MCM3AP-AS1 promotes the activity of CRC cells by activating VEGF/VEGFR2.

In follow-up research, we will also study the regulatory impact of MCM3AP-AS1 on downstream target genes in CRC and construct a tumor-bearing nude mouse model to confirm the impacts of MCM3AP-AS1 on specific tumorigenesis. In addition, research subjects need to be followed up for a longer period to confirm the impacts of MCM3AP-AS1 on the long-term prognosis of CRC patients. In summary, MCM3AP-AS1 overexpression in CRC implies an increased risk of an unfavorable prognosis and intensifies the invasiveness and proliferation of CRC cells by activating the VEGF/VEGFR2 signaling pathway.

## Figures and Tables

**Figure 1:** qRT–PCR was used to detect the expression level of MCM3AP-AS1 in the blood of CRC patients and healthy persons. (a) Comparison of MCM3AP-AS1 between CRC patients and healthy individuals. The MCM3AP-AS1 level of CRC patients was significantly higher than that of healthy persons. Comparison between the two groups #*P* < 0.05. (b) ROC curve of MCM3AP-AS1 for predicting CRC occurrence. “#” indicates *P* < 0.05 for the comparison between the two groups.

**Figure 2:** Prognostic value of MCM3AP-AS1. (a) MCM3AP-AS1 in CRC patients before and after therapy. The expression level of MCM3AP-AS1 in CRC patients after treatment was lower than that before treatment. (b) MCM3AP-AS1 in the patients who died and those who survived. The expression level of MCM3AP-AS1 in patients who died after treatment was higher than that in patients who survived. (c) MCM3AP-AS1 in patients with recurrence and those without recurrence. (d) ROC of MCM3AP-AS1 after therapy in forecasting death. The expression level of MCM3AP-AS1 in patients with prognostic recurrence after treatment was higher than that in patients without recurrence. (e) ROC of MCM3AP-AS1 after therapy in forecasting recurrence. (f) Survival curve of the high and low MCM3AP-AS1 expression groups. The prognostic mortality rate of the high MCM3AP-AS1 expression group was higher than that of the low MCM3AP-AS1 expression group. Comparison between the two groups #*P* < 0.05.

**Figure 3:** Analysis of MCM3AP-AS1 based on the database. (a) Expression analysis of MCM3AP-AS1 in other tumor diseases. (b) Prognostic analysis of MCM3AP-AS1.

**Figure 4:** The effect of MCM3AP-AS1 silencing on the proliferation and invasion of CRC cells. (a) The expression of MCM3AP-AS1 in HCT116, SW480, and CCD-18Co cells. (b) Growth curve of HCT116 cells. (c) Growth curve of SW480 cells. (d) Results of Transwell experiments. (e) The number of invading cells. Comparison between the two groups #*P* < 0.05.

**Figure 5:** The effect of MCM3AP-AS1 silencing on CRC cell apoptotic proteins. (a) Western blot map of HCT116 cells. (b) Apoptosis-associated proteins in HCT116 cells. (c) Western blot map of SW480 cells. (d) Apoptosis-associated proteins in SW480 cells. Comparison between the two groups #*P* < 0.05.

**Figure 6:** Impacts of MCM3AP-AS1 on the VEGF/VEGFR2 pathway. (a) qRT–PCR was used to detect the levels of VEGF and VEGFR2 mRNA in HCT116, SW480, and CCD-18Co cells. (b) qRT–PCR was used to detect the effect of MCM3AP-AS1 on the VEGF/VEGFR2 pathway in HCT116 cells. (c) qRT–PCR was used to detect the effect of MCM3AP-AS1 on the VEGF/VEGFR2 pathway in SW480 cells. (d) Western blot map of HCT116 cells. (e) Western blot detection of the effect of MCM3AP-AS1 on the VEGF/VEGFR2 pathway in HCT116 cells. (f) Western blot map of SW480 cells. (g) Western blot detection of the effect of MCM3AP-AS1 on the VEGF/VEGFR2 pathway in SW480 cells. Comparison between the two groups #*P* < 0.05.

**Figure 7:** The effect of inhibiting the VEGF/VEGFR2 pathway on the proliferation and invasion of CRC cells. (a) Growth curve of HCT116 cells. (b) Growth curve of SW480 cells. (c) Results of Transwell experiments. (d) The number of invaded cells. Comparison between the two groups #*P* < 0.05.

**Figure 8:** The effect of inhibiting the VEGF/VEGFR2 pathway on apoptotic proteins in CRC cells. (a) Western blot map of HCT116 cells. (b) Apoptosis-associated proteins in HCT116 cells. (c) Western blot map of SW480 cells. (d) Apoptosis-associated proteins in SW480 cells. Comparison between the two groups #*P* < 0.05.

**Table 1:** Primer sequences.

Molecule	F (5′-3′)	R (5′-3′)
MCM3AP-AS1	GCTGCTAATGGCAACACTGA	AGGTGCTGTCTGGTGGAGAT
GAPDH	CAGGAGGCATTGCTGATGAT	GAAGGCTGGGGCTCATTT
VEGF	CGAGACGCAGCGACAAGGCA	ACCTCTCCAAACCGTTGGCACG
VEGFR2	TTTGGCAAATACAACCCTTCAGA	GCAGAAGATACTGTCACCACC
*β*-Actin	CTGAAGGTCAAAGGGAAT	CAGAGTCTTGATGATCTC

## Data Availability

Readers can obtain the data upon request to the corresponding authors.
